The article "Evaluation of Cardiac Function of Pregnant Women with High Blood Pressure during Gestation Period and Coupling of Hearts with Peripheral Vessels by Ultrasonic Cardiogram under Artificial Intelligence Algorithm" was retracted in 2023. Reasons: signs of a paper mill; compromised peer review; unreliable results or conclusions.

# Evaluation of Cardiac Function of Pregnant Women with High Blood Pressure during Gestation Period and Coupling of Hearts with Peripheral Vessels by Ultrasonic Cardiogram under Artificial Intelligence Algorithm

**DOI:** 10.1155/2022/5019153

**Published:** 2022-01-27

**Authors:** Xia Zhang, Xi Liang, Wen Cao

**Affiliations:** Department of Function, The Affiliated Wuxi Maternal and Child Health Care Hospital of Nanjing Medical University, Wuxi, 214002 Jiangsu, China

## Abstract

The research was aimed at analyzing the value of the optimized eXtreme Gradient Boosting (XGBoost) algorithm-based ultrasound cardiogram images in the diagnosis of pregnant hypertension patients. A total of 145 pregnant women (85 cases suffered from hypertension disease during pregnancy and 60 other normal women were healthy) were selected as the reference to the comparison and analysis of ultrasound cardiac function parameter, common carotid artery parameter, and the coupling relationship between hearts and cervical vessels of pregnant hypertension patients. The results demonstrated ultrasound cardiac function parameter of pregnant hypertension patients as follows. The maximum volume of the left atrium (LAVmax) was 35.65 mm, left ventricular end-systolic volume (LVESV) was 31.07 mm, and left ventricular end-diastolic volume (LVEDV) was 88.73 mm. All the above indexes were obviously higher than those of the normal control group (*P* < 0.05). Besides, intima-media thickness (IMT) of common carotid artery (465.84 *μ*m), pulse wave velocity (PWV) (8.09 m/s), pressure of turning point 1 from isovolumic contraction phase to ejection phase (PT1) (126.5 mmHg), arterial enhancement pressure (AP) (6.14 mmHg), and arterial pressure enhancement index (8.58%) were all significantly higher than those of the normal control group (*P* < 0.05). In addition, the correlation between the coupling (*E*/*A*) of hearts and carotid artery of pregnant hypertension patients and PWV was not obvious (*r* = −0.08432, *P* > 0.05). The results of the research indicated that intima-media inside carotid artery of pregnant hypertension patients thickened obviously, and it became less elastic compared with that of normal healthy pregnant women. What is more, cardiac morphological changes were manifested mainly as the enlargement of the left atrial chamber and the thickening of the interventricular septum. Volume load and blood flow velocity both increased, and left ventricular diastolic function was damaged. XGBoost algorithm-based ultrasound cardiogram images could improve the diagnostic effects of hypertension during pregnancy effectively.

## 1. Introduction

Pregnancy is a special physiological state. In this period, every system throughout pregnant women's body underwent a series of changes to promote fetuses' growth and development. The changes in cardiovascular system are especially obvious [1]. Hypertensive disorder complicating pregnancy (HDCP) is a kind of common and severe complication appearing only during pregnancy. According to related statistics, the current incidence of this disease accounted for 5%-10% among all pregnant women, which was a major cause of death of pregnant women [2]. According to epidemiological data, it was shown that HDCP was caused by multiple factors affecting each other, and this symptom would potentially result from many other factors, such as pregnant women's age, the number of pregnancies, familial inheritance history, nutritious condition, social and economic status, physical activities they engage in, and neuroendocrine [3, 4]. However, the exact pathogenesis is unknown now, which causes great difficulty in clinical prevention.

The article "Evaluation of Cardiac Function of Pregnant Women with High Blood Pressure during Gestation Period and Coupling of Hearts with Peripheral Vessels by Ultrasonic Cardiogram under Artificial Intelligence Algorithm" was retracted in 2023. Reasons: signs of a paper mill; compromised peer review; unreliable results or conclusions.

Related studies demonstrated that the pathological changes of hypertension during pregnancy of patients were caused mainly by arteriolar spasm throughout the body, which resulted in the changes of systemic hemodynamics. Its main change was the change of stiffness of vessel walls [5]. Pathological studies confirmed that the impact force and mechanical pressure exerted on body vessel walls by blood flow caused vascular endothelial injury when blood pressure was enhanced. At the same time, blood flow dysfunction occurred, which stiffened blood walls. Based on the stiffening of blood walls, small artery walls stiffened and acute arteriosclerosis and thromboembolism occurred in blood in the myometrium and decidual layer [6]. With profound studies in recent years, it was pointed out that blood vessel stiffening of hypertension patients during pregnancy could last until about 4 weeks after parturition. During pregnancy, blood pressure was enhanced constantly, which increased cardiac preload. Cardiac function of patients with hypertensive disorder complicating pregnancy (HDCP) was changed with various degrees with the severity of disease. Real-time monitoring of cardiac function was likely to become an effective method of reflecting the severity of disease of patients objectively [7, 8]. There were a large number of fundamental research into the changes in cardiac structure and function of hypertension patients during pregnancy, but the reports on whether peripheral elastic blood vessels were abnormal, such as carotid artery, were rare. Besides, the coupling function of heart and peripheral blood vessels was unknown. The decrease in elasticity of artery was the pathological condition and main factor of the occurrence of cardiovascular disease. Arterial stiffness could be viewed as the relationship between geometric shape blood vessel walls and the blood pressure of pulse exerting on blood vessel walls when arterial diameter was changed. The correlation between blood pressure and arterial diameter is related to the elasticity of arterial walls. In the process of pregnancy as long as 9 months, the heart burden of some pregnant women was gradually increasing, which might cause HDCP and other complications [9, 10]. Therefore, it was imperative to assess the relationship between the elasticity of peripheral blood vessels and cardiac function during pregnancy.

The article "Evaluation of Cardiac Function of Pregnant Women with High Blood Pressure during Gestation Period and Coupling of Hearts with Peripheral Vessels by Ultrasonic Cardiogram under Artificial Intelligence Algorithm" was retracted in 2023. Reasons: signs of a paper mill; compromised peer review; unreliable results or conclusions.

In terms of previous assessment methods of arterial structure, some imaging methods, such as computerized tomography (CT) and magnetic resonance imaging (MRI), were adopted to assess intima-media thickness (IMT) of carotid artery. Then, the blood pressure ratio between the ankle and arm was obtained based on the blood pressure values of body upper arm and ankle, which is called ankle-brachial index (ABI) [11]. Nevertheless, the above method was not suitable for pregnant women examination because radiation was generated in imaging examination and pressure needed to be applied to limbs before ABI was obtained. In contrast, artificial intelligence- (AI-) based ultrasound cardiogram images could obtain blood vessel IMT data and related data on blood vessel elasticity with no pressure. The accuracy of data extraction is verified by related studies [12]. XGBoost algorithm is widely adopted in data mining and recommendation system recently. Hence, it is utilized in the research to evaluate the cardiac function state of HDCP patients and its coupling with peripheral blood vessels with its high efficiency and flexibility. The advantages of ultrasound cardiogram images are made use of to conduct the research, such as convenience and nontrauma. The evaluation in this research offered certain theoretical help to the diagnosis and treatment of clinical pregnant hypertension patients.

## 2. Materials and Methodology

### 2.1. General Data

From August 2018 to March 2020, a total number of 145 pregnant women who experienced regular prenatal check in hospital were chosen as the research objects. Among these patients, 85 pregnant women with high blood pressure were in the experimental group while the other 60 healthy pregnant women were in the control group. The criteria of selecting pregnant patients with high blood pressure included (a) patients who met the diagnostic standard of high blood pressure disease during pregnancy, which was the constant increase of blood pressure 20 weeks before or prior to pregnancy, reaching or even greater than 140/90 mmHg; (b) patients with singleton pregnancy; and (c) patients who had diseases affecting the blood pressure level of human body, such as combined hyperthyroidism and pheochromocytoma. Exclusion criteria were as follows: (a) patients with basic heart disease before pregnancy; (b) patients with gestational diabetes mellitus, heart disease, and other complications during pregnancy; and (c) patients who had some systemic infectious complications. Patients in the research and their family members were informed and signed the informed consent form. Besides, this study was approved by the ethics committee of the hospital.

The article "Evaluation of Cardiac Function of Pregnant Women with High Blood Pressure during Gestation Period and Coupling of Hearts with Peripheral Vessels by Ultrasonic Cardiogram under Artificial Intelligence Algorithm" was retracted in 2023. Reasons: signs of a paper mill; compromised peer review; unreliable results or conclusions.

### 2.2. Apparatus and Methods

Esaote color Doppler ultrasonic diagnostic apparatus (Mylab70XV, LA523 searching unit, 4-13 MHz) was used. The assessment of ultrasonic cardiac function parameters was as follows: the state of heart function of patients in the experimental and control groups was tested by color Doppler ultrasonic diagnostic apparatus immediately after being admitted to the hospital. Firstly, the searching unit was put at the apex part of the patients' heart and patients were asked to hold their breath, during which the position of the unit was adjusted to get the standard image of four chambers in the patients' hearts. After this, the image of the intima in the left atrium and related data were described and recorded. Finally, maximum volume of the left atrium (LAVmax), left ventricular end-systolic volume (LVESV), and the value of left ventricular end-diastolic volume (LVEDV) were all obtained. The method of measuring IMT in blood vessels and the elasticity index was that patients should lie on their backs and then rest silently for five minutes. In this period, the common carotid artery was presented and its image was acquired. All images were optimized by adopting XGBoost algorithm.

### 2.3. XGBoost Algorithm Principle

Extreme gradient boosting algorithm, also called eXtreme gradient boosting (XGBoost), is one of the improved boosting algorithms, and its principle can be explained as a strong classifier attained by the concentration and synthesis of many weak classifiers. XGBoost can be seen as a kind of the improved tree-shaped model of a new stronger classifier, which is generated by gathering and synthesizing lots of decision-making trees. Also, XGBoost belongs to integrated algorithms.

XGBoost made use of classification and regression tree (CART) model, which assumed that the tree was transformed into a binary tree by keeping splitting features. It was assumed that the current node of CART was the manipulation over the direction of this tree by the *m*th eigenvalue, and the samples of the eigenvalues less than *n* were viewed as left subtrees, while those greater than *n* were regarded as right subtrees. In this way, the first equation was obtained.

(1) $$\begin{array}{c} R_{1}\left(m,n\right)=\left\{z\right|z^{\left(m\right)}\leq \left.n\right\},\\ R_{2}\left(m,n\right)=\left\{z\right|z^{\left(m\right)}\geq \left.n\right\}. \end{array}$$

The essence of CART's regression to the tree is that sample space was divided within this characteristic dimension, and the optimization of the division of sample space was a nondeterministic issue with polynomial complexity. Therefore, heuristic method was used to tackle with the problem in decision-making tree model. The function generated by the typical CART is shown below.

(2) $$\begin{array}{c} \underset{z_{i}\in R_{S}}{\sum }{\left(y_{i}-f\left(z_{i}\right)\right)}^{2}. \end{array}$$

Consequently, optimal segmentation characteristic value and the function corresponding to optimal segmentation point *n* people calculated could be used to solve the following function:

(3) $$\begin{array}{c} f_{z,y}=\underset{m,n}{\min}\left[\underset{c_{1}}{\min}\right.\underset{z_{i}\in R_{1}\left(m,n\right)}{\sum }{\left(y_{i}-c_{1}\right)}^{2}+\underset{c_{2}}{\min}\underset{z_{i}\in R_{2}\left(m,n\right)}{\sum }\left(y_{i}-c_{2}\right)\left.{}^{2}\right]. \end{array}$$

As a result, people could acquire optimal segmentation characteristic and optimal segmentation point by viewing all segmentation points of all characteristics. The final result would be the transformation into a regression tree.

The article "Evaluation of Cardiac Function of Pregnant Women with High Blood Pressure during Gestation Period and Coupling of Hearts with Peripheral Vessels by Ultrasonic Cardiogram under Artificial Intelligence Algorithm" was retracted in 2023. Reasons: signs of a paper mill; compromised peer review; unreliable results or conclusions.

Keeping adding trees is the principle of XGBoost algorithm. To be specific, trees were generated one after another by constant split of characteristics. In essence, the appearance of each new tree is fitting the residual caused by the previous prediction by obtaining a new objective function. Once people got *q* trees after continuous training, they would predict the score of a sample. In fact, there would be a leaf node corresponding to each tree and a corresponding score for every leaf node according to the features of samples. At the end, the predicted value of samples would be acquired only if the corresponding score of each tree was added.

The objective function of XGBoost was defined as follows:

(4) $$\begin{array}{c} \text{Obm}=\overset{e}{\underset{i=1}{\sum }}\text{l}\left(y_{i},{\overset{⌢}{y}}_{i}\right)+\overset{Q}{\underset{q=1}{\sum }}\Omega \left(f_{q}\right). \end{array}$$

The above objective function consists of two components, one of which is used to evaluate the gap between the predicted score and the true score. Regularization item is another component. Apart from the objective function, regularization item is also made up of two components, including the number of leaf nodes (shown as *A*) and the score of leaf nodes (shown as *w*). Γ can regulate the number of leaf nodes, and *λ* can regulate leaf nodes to avoid its score becoming too large, which can prevent overfitting.

The article "Evaluation of Cardiac Function of Pregnant Women with High Blood Pressure during Gestation Period and Coupling of Hearts with Peripheral Vessels by Ultrasonic Cardiogram under Artificial Intelligence Algorithm" was retracted in 2023. Reasons: signs of a paper mill; compromised peer review; unreliable results or conclusions.

As stated above, fitting the residual appearing in the previous prediction is necessary for the new tree. In other words, the predicted score could be expressed by

(5) $$\begin{array}{c} {{\overset{⌢}{y}}_{i}}^{\left(a\right)}={{\overset{⌢}{y}}_{i}}^{\left(a-1\right)}+f_{a}\left(z_{i}\right). \end{array}$$

Meanwhile, the objective function could be rewritten as

(6) $$\begin{array}{c} \partial^{\left(a\right)}=\overset{e}{\underset{i=1}{\sum }}\text{l}\left(y_{i},{{\overset{⌢}{y}}_{i}}^{\left(a-1\right)}+f_{a}\left(z_{i}\right)\right)+\Omega \left(f_{a}\right). \end{array}$$

Apparently, the next step was to find *f*_*a*_ that could minimize the objective function. The idea of XGBoost was to approximate it using the Taylor second-order expansion at *f*_*a*_ = 0. Therefore, the objective function was approximated as

(7) $$\begin{array}{c} \partial^{\left(a\right)}≃\overset{e}{\underset{i=1}{\sum }}\left[\text{l}\right.\left(y_{i},{{\overset{⌢}{y}}_{i}}^{\left(a-1\right)}\right)+d_{i}f_{a}\left(z_{i}\right)+\frac{1}{2}j_{i}f_{a}^{2}\left.\left(z_{i}\right)\right]+\Omega \left(f_{a}\right). \end{array}$$

In the above equation, *d*_*i*_ referred to first-order derivative and *j*_*i*_ meant second-order derivative, both of which could be calculated in

(8) $$\begin{array}{c} d_{i}=\gamma_{{\overset{⌢}{y}}^{\left(a-1\right)}}\text{l}\left(y_{i},{{\overset{⌢}{y}}_{i}}^{\left(a-1\right)}\right),\\ j_{i}={\gamma_{{\overset{⌢}{y}}^{\left(a-1\right)}}}^{\bar{2}}\text{l}\left(y_{i},{{\overset{⌢}{y}}_{i}}^{\left(a-1\right)}\right). \end{array}$$

The predicted score and the residual of *y* caused no effect on the optimization of the objective function, so they could be deleted directly. The objective function was presented as

(9) $$\begin{array}{c} \partial^{\left(a\right)}=\overset{e}{\underset{i=1}{\sum }}\left[d_{i}\right.f_{a}\left(z_{i}\right)+\frac{1}{2}j_{i}f_{a}^{2}\left.\left(z_{i}\right)\right]+\Omega \left(f_{a}\right). \end{array}$$

The equation was obtained by adding the missing function values of each sample. Based on the above content, each sample would fall into a leaf node, so people could combine the samples of all same leaf nodes; the process of which was demonstrated in

(10) $$\begin{array}{c} {\text{Obm}}^{\left(a\right)}≃\overset{e}{\underset{i=1}{\sum }}\left[d_{i}\right.f_{a}\left(z_{i}\right)+\frac{1}{2}j_{i}f_{a}^{2}\left.\left(z_{i}\right)\right]+\Omega \left(f_{a}\right)=\overset{e}{\underset{i=1}{\sum }}\left[d_{i}\right.f_{a}\left(z_{i}\right)+\frac{1}{2}j_{i}f_{a}^{2}\left.\left(z_{i}\right)\right]+\alpha A+\lambda \frac{1}{2}\overset{A}{\underset{m=1}{\sum }}w_{m}^{2}=\overset{A}{\underset{m=1}{\sum }}\left[\left(\underset{i\in I_{m}}{\sum }d_{i}\right)w_{m}\right.+\frac{1}{2}\left(\underset{i\in I_{m}}{\sum }j_{i}+\lambda \right)\left.w_{m}^{2}\right]+\alpha A. \end{array}$$

Therefore, the objective function could be rewritten as a quadratic function of one variable involving the score of leaf nodes (*w*) in the above equation. In this equation, it was easy to figure out the values of optimal *w* and the objective function, which could be achieved by using vertex equation. Hence, optimal *w* value and the equation of the objective function are shown as equations (11) and (12), respectively:

(11) $$\begin{array}{c} {w_{m}}^{*}=-\frac{M_{m}}{J_{m}+\lambda }, \end{array}$$

(12) $$\begin{array}{c} \text{Obm}=-\frac{1}{2}\overset{A}{\underset{m=1}{\sum }}\frac{{M_{m}}^{2}}{J_{m}+\lambda }+\alpha A. \end{array}$$

The gain equation of XGBoost was expressed as

(13) $$\begin{array}{c} L_{\text{split}}=\frac{1}{2}\left[\frac{{M_{L}}^{2}}{J_{L}+\lambda }\right.+\frac{{M_{R}}^{2}}{J_{R}+\lambda }-\left.\frac{{\left(M_{L}+M_{R}\right)}^{2}}{J_{L}+J_{R}+\lambda }\right]-\gamma . \end{array}$$

The article "Evaluation of Cardiac Function of Pregnant Women with High Blood Pressure during Gestation Period and Coupling of Hearts with Peripheral Vessels by Ultrasonic Cardiogram under Artificial Intelligence Algorithm" was retracted in 2023. Reasons: signs of a paper mill; compromised peer review; unreliable results or conclusions.

### 2.4. Modelling Procedure by XGBoost

The modelling process by XGBoost algorithm was explained as follows.

Input: training dataset *D* = {(*z*_1_, *y*_1_), (*z*_2_, *y*_2_), ⋯, (*z*_*n*_, *y*_*n*_)}; *A* that represented the number of the iteration of weak classifiers was input and weak classifiers were CART used in the research. In the equation, *z* and *y* were samples and true labels matched by samples, respectively.

Output: strong classifier *f*(*z*).

For each weak classification learner *M*,

1. browse through each characteristic *q*
2. view every *z*_*mq*_ under the current feature *q*. Front node samples were divided into left and right subtrees by the split eigenvalues. Based on the equation, information gain was figured out, and then, the features and feature splitting values corresponding to the maximum information gain were selected to split nodes. When the maximum value of left subtrees (*L*_split_) became less than 0, the splitting ceased. Γ could be seen as the split threshold that possessed the function of prepruning. The node splitting needed to be repeated. Optimal splitting value could be found out by scanning from left to right in the order of eigenvalues

### 2.5. Observation Indexes

Ultrasound cardiac function parameters of patients in two groups were observed and compared, including LAVmax, LVESV, and LVEDV. Besides, the cardiac chambers and pericardium ultrasound images of patients in two groups before and after XGBoost algorithm optimization were also observed and compared. In terms of carotid artery parameters, IMT, pulse wave velocity (PWV), pressure of turning point 1 from isovolumic contraction phase to ejection phase (PT1), arterial enhancement pressure (AP), and augmentation index (AIx) were observed, and the coupling relationship between hearts and cervical blood vessels of pregnant hypertension patients was analyzed.

The article "Evaluation of Cardiac Function of Pregnant Women with High Blood Pressure during Gestation Period and Coupling of Hearts with Peripheral Vessels by Ultrasonic Cardiogram under Artificial Intelligence Algorithm" was retracted in 2023. Reasons: signs of a paper mill; compromised peer review; unreliable results or conclusions.

### 2.6. Statistical Analysis

All data obtained by this work was analyzed and processed by Statistical Product and Service Solutions (SPSS) software in version 23.0, and measurement data passed the normality test and were manifested at the form of *x* ± *s*. Data from several groups were compared by adopting one-way analysis of variance method, while *q* test was used for data comparison between two groups. As to the correlation analysis, Pearson-related test was involved and correlation coefficient *r* was calculated using the Spearman rank correlation. When *P* was less than 0.05, it was implied that the difference had statistical meaning.

## 3. Results

Table 1 presents general data on patients in the experimental group and the control group included in the research.

The differences of data on age and average pregnancy weeks between pregnant women in two groups had no statistical meaning, and *P* > 0.05.

### 3.1. Ultrasonic Heart Function Parameters

- The comparison of ultrasonic heart function parameters between patients in the experimental groups and from the control groups, including the indexes of LAVmax, LVESV, and LVEDV, is shown in Figure 1.

Figure 1 shows that the indexes of pregnant patients with high blood pressure, including LAVmax, LVESV, and LVEDV, were all greater than those of patients in the control group. The differences of ultrasonic heart function parameter level between patients in two groups had statistical significance (*P* < 0.05).

(b) Heart chambers and echocardiogram of patients in two groups are shown in Figures 2–4, respectively.

Figures 2–4 indicate that the left atriums and left chambers of pregnant patients with high blood pressure were obviously bigger than those of patients in the control group (*P* < 0.05). This difference was statistically significant. Meanwhile, some indexes, including LA diameter, interventricular septal diameter (IVSd), and LVEDD, were all apparently greater than those of patients in the control group (*P* < 0.05), which also reflected statistical meaning.

(c) Tissue Doppler showed the ratios of left ventricular front wall and side wall *E*/*A* and of blood flow velocity *E* during color Doppler mitral systole and tissue Doppler left ventricular front wall and side wall *e* (*E*/front wall *e* and *E*/side wall *e*); both of which are demonstrated in Figure 5.

The article "Evaluation of Cardiac Function of Pregnant Women with High Blood Pressure during Gestation Period and Coupling of Hearts with Peripheral Vessels by Ultrasonic Cardiogram under Artificial Intelligence Algorithm" was retracted in 2023. Reasons: signs of a paper mill; compromised peer review; unreliable results or conclusions.

Figure 5 reveals that the left ventricular anterior wall and side wall *E*/*A* in tissue Doppler of pregnant patients with high blood pressure were significantly less than those of patients in the control group (*P* < 0.05). Besides, the ratio of blood flow velocity *E* during color Doppler mitral systole and tissue Doppler left ventricular front wall and side wall *e* (*E*/front wall *e* and *E*/side wall *e*) was evidently greater than that in the control group (*P* < 0.05). The difference had statistical meaning.

### 3.2. Common Carotid Artery Parameters

IMT in common carotid arteries, PWV, PT1 from isovolumic systole to ejection period, augmented pressure (AP) on arteries, and augmentation index (AIx) of artery pressure of patients in two groups are shown in Figures 6 and 7.

Figures 6 and 7 show that IMT in common carotid arteries, PWV, PT1 from isovolumic systole to ejection period, AP on arteries, and AIx of artery pressure of pregnant patients with high blood pressure in the experimental group were all obviously greater than those of patients in the control group (*P* < 0.05). This difference had statistical significance.

### 3.3. The Coupling Relationship between Hearts and Cervical Vessels of Pregnant Patients with High Blood Pressure

The coupling relationship between hearts and cervical vessels of pregnant patients with high blood pressure is presented in Figure 8.

Figure 8 indicates that the correlation between *E*/*A* and PWV was not very apparent (*r* = −0.08432, *P* > 0.05).

## 4. Discussion

Clinical ultrasonic cardiogram was applied in auxiliary diagnosis of high blood pressure during pregnancy, and the research of the application value of auxiliary diagnosis of high blood pressure during pregnancy by the imagological features of ultrasonic cardiogram, which was based on XGBoost algorithm, was the hot issue on the research about imagology [13]. It was pointed out in related literature that the diagnosis of diseases and the investigation into the severity of diseases using some technologies at earlier stage could improve the high-quality diagnostic effect in later stage. The obvious increase in blood pressure increased pump load of the left heart and caused the changes of myocardial cells in patients' body, which led to problems in systolic and diastolic functions of the left heart. As a result, cardiac failure appeared [14, 15]. This phenomenon was consistent with the result of this research. In this research, the left heart function parameter indexes of pregnant patients with high blood pressure and normal pregnant women were evaluated by ultrasonic cardiogram, which indicated that the left heart parameters of pregnant patients with high blood pressure, including LAVmax, LVESV, and LVEDV, all rose obviously compared with those in the control group (*P* < 0.05). There was a statistical significance in this difference, which showed that dysfunction really existed in the left heart of pregnant patients with high blood pressure.

The article "Evaluation of Cardiac Function of Pregnant Women with High Blood Pressure during Gestation Period and Coupling of Hearts with Peripheral Vessels by Ultrasonic Cardiogram under Artificial Intelligence Algorithm" was retracted in 2023. Reasons: signs of a paper mill; compromised peer review; unreliable results or conclusions.

The change in the pressure on arteries was crucial for and even played a decisive role in the stiffness of blood vessels in arteries. Meanwhile, it was also an independent factor in predicting the occurrence of cardiovascular diseases and the organic damage. Related literature showed that IMT in carotid arteries was a key indicator reflecting whether earlier artery walls deteriorate. The damage caused by the increase of IMT resulted from the long-term influence of high-risk factors on artery walls, one of which was probably the rise of blood pressure of patients during pregnancy. If mean artery pressure (MAP) was equal to or greater than 85 mmHg, it was possible that patients would suffer from preeclampsia. If MAP was equal to or greater than 140 mmHg, cerebrovascular disease was likely to occur, which would make pregnant patients fall into a coma and even lose their lives [16, 17]. The values of MAP of all pregnant patients with high blood pressure researched in this study were all greater than 85 mmHg, and IMT was obviously greater than those in the control group. The results demonstrated that the blood vessels of pregnant patients with high blood pressure also became relatively less elastic, and the blood stiffness indexes, such as PWV, T1, and AIx, all increased significantly (*P* < 0.05). The difference had statistical meaning. High blood pressure weakened the function of vascular endothelium of patients and vascular elasticity. What is more, it caused a great increase in the possibility of atherosclerosis in the future. PWV, a significant indicator associated firmly with high-risk factors of causing cardiovascular disease, had a much more superior predicative function of the possibility of cardiovascular disease than that of patients' age, gender, the value of blood pressure, and cognitive capacity [18]. The pulse wave was generated by the diffusion of heart impulse along arteries and flowing blood toward surrounding, which caused the changes in the pressure on vascular wall, blood flow velocity, and vascular wall volume. These changes could be detected by different receptors. The diameter of arterial blood vessels, the thickness of vessel walls, and the elasticity of arterial walls were the main factors in determining PWV. To be specific, relatively more elastic arterial blood vessels meant thinner intima- media and lower PWV [19]. The research found out that thicker intima-media of carotid arteries of pregnant patients with high blood pressure meant higher PWV, which showed an obvious tendency in arterial stiffening. When the atherosclerosis of women with pregnancy complications was evaluated, PWV showed higher accuracy than artery pressure. According to relevant data, PWV positively correlated with arterial pressure. Ma et al. [20] proved that there was a significant relevance between PWV of patients with primary hypertension and prognosis of cardiovascular disease caused by multiple factors by multifactor regression analysis method. However, whether this relevance could also be found in pregnant patients with high blood pressure needed to be verified. AP and AIx could be used to predict the early changes in the function of artery, which indicated the tendency of arterial stiffening and reflective wave intensification. AIx was another essential factor that implied the degree of arterial compliance, which was primarily determined by the elasticity and the diameter of the walls of peripheral arterioles. These two factors determined where the reverse reflective waves fell down in diastolic or systolic period. As average pressure on arteries grew, AIx also increased. Greater AIx value showed a low degree of arterial compliance [21, 22]. Another research finding was the significant rise of AIx of pregnant patients with high blood pressure, which further illustrated that the vascular stiffness of pregnant patients with high blood pressure went up obviously.

The article "Evaluation of Cardiac Function of Pregnant Women with High Blood Pressure during Gestation Period and Coupling of Hearts with Peripheral Vessels by Ultrasonic Cardiogram under Artificial Intelligence Algorithm" was retracted in 2023. Reasons: signs of a paper mill; compromised peer review; unreliable results or conclusions.

It was found out in related research that the changes in cardiac morphology of patients with severe high blood pressure at the later stage of pregnancy mainly included hydropericardium, LA chamber expansion, and interventricular septum thickening, which caused damage to diastolic function of the left heart chamber. It was reported that the weakening of diastolic function of the left heart chamber preceded over that of systolic function for patients with preeclampsia [23]. The blood pressure of pregnant patients with high blood pressure kept rising 20 weeks after pregnancy, which led to the increases of left ventricular afterload, LA chamber expansion, and interventricular septum compensatory hypertrophy. The weakening of the elasticity of the left heart chamber resulted in the inadequacy in diastolic functions of the left heart chamber, which were manifested mainly by the diastole of the left heart chamber and filling obstruction. The proportion of filling in the left heart chamber was increased by atrial systole [24, 25]. The change in blood flow in the mitral valve was mainly the reduction of peak *E* and the increase of peak *A*, namely, *E*/*A* < 1. In the experiment, 40 patients were featured with *E*/*A* > 1, 26 of which were characterized by *E*/*A* < 1 for front walls and for side walls in the left heart chambers. The number of patients with *E*/*A* < 1 was 17, whose *E*/*A* of both front walls and side walls of the left heart chambers were less than 1; the *E*/*A* value of two patients was greater than 2, which might be caused by the obvious weakening of the compliance of the left heart chamber, which referred to the failure of filling pressure to increasing along with left heart chamber expansion. The clinical manifestation of this feature was the increase of filling pressure at earlier diastolic stage, which resulted in the enhancement of peak *E*. At later diastolic stage of the left heart chamber, filling pressure rose so that ventricular filling rate decreased during atrial contraction and peak *A* weakened, even disappeared [26]. Based on related experiments, it was proved that the correlations between the damage of diastolic function of pregnant patients with high blood pressure and the change in vascular wall elasticity existed, but they were not closely related, which might be due to the limited left ventricular filling of some patients or the insufficiency of cases in the experimental group or the difference in the severity of high blood pressure of pregnant patients. Further research needed to be focused on the coupling of cardiovascular vessels of pregnant patients with high blood pressure.

The article "Evaluation of Cardiac Function of Pregnant Women with High Blood Pressure during Gestation Period and Coupling of Hearts with Peripheral Vessels by Ultrasonic Cardiogram under Artificial Intelligence Algorithm" was retracted in 2023. Reasons: signs of a paper mill; compromised peer review; unreliable results or conclusions.

## 5. Conclusion

XGBoost algorithm optimization-based ultrasound cardiogram images were adopted to examine and diagnose pregnant hypertension patients in this research. The results of analysis found out that XGBoost algorithm could obtain clearer and more accurate cardiogram images and data of patients quickly and effectively. Compared with normal healthy pregnant women, IMT in carotid artery increased obviously and intima-media became less elastic. The enlargement of the left atrial chamber and the thickening of the interventricular septum were the main changes of cardiac morphology. What is more, cardiac volume load and blood flow velocity both increased, which caused damage to left ventricular diastolic function. Ultrasound cardiogram images under XGBoost algorithm could obtain blood vessel IMT data and data related to blood vessel elasticity, which improved the diagnostic accuracy of hypertension during pregnancy effectively.

## Figures and Tables

**Figure 1:** Ultrasonic heart function parameters of patients in two groups (∗# represented *P* < 0.05, and the differences showed statistical meaning).

The article "Evaluation of Cardiac Function of Pregnant Women with High Blood Pressure during Gestation Period and Coupling of Hearts with Peripheral Vessels by Ultrasonic Cardiogram under Artificial Intelligence Algorithm" was retracted in 2023. Reasons: signs of a paper mill; compromised peer review; unreliable results or conclusions.

**Figure 2:** (a) The left atriums and left chambers of pregnant patients with high blood pressure were relatively big, and pericardial effusion was detected (before the optimization of XGBoost algorithm) (the arrow in (a) referred to pericardial effusion). (b) The left atriums and left chambers of pregnant patients with high blood pressure were relatively big, and pericardial effusion was detected (after the optimization of XGBoost algorithm) (the arrow in (b) referred to pericardial effusion).

**Figure 3:** (a) The size of the atriums and heart chambers of patients in the control group was normal, and there was no pericardial effusion (before the optimization of XGBoost algorithm). (b) The size of the atriums and heart chambers of patients in the control group was normal, and there was no pericardial effusion (after the optimization of XGBoost algorithm).

**Figure 4:** The comparison of cardiac shape LA diameter, interventricular septal thickness, and LVEDD between two groups (∗# represented *P* < 0.05, and the differences showed statistical meaning).

**Figure 5:** The ratios of left ventricular front wall and side wall *E*/*A* and of blood flow velocity *E* during mitral systole and tissue Doppler left ventricular front wall and side wall *e* (∗# represented *P* < 0.05, and the differences showed statistical meaning).

**Figure 6:** PT1 and AP on arteries (∗# represented *P* < 0.05, and the differences showed statistical meaning).

**Figure 7:** IMT in common carotid arteries, PWV, and AIx of artery pressure of patients in two groups (∗# represented *P* < 0.05, and the differences showed statistical meaning).

**Figure 8:** The coupling relationship between hearts and cervical arteries of pregnant patients with high blood pressure (*r* = 0.08432, *P* > 0.05).

**Table 1:** General data on patients in two groups ($\bar{x}\pm s$).

Indexes	Average age (years old)	Average pregnancy week (weeks)	Average body mass index (kg/m^2^)
Pregnant hypertension women (*n* = 85)	27.35 ± 3.85	33.43 ± 4.67	26.28 ± 2.67
Normal healthy women (*n* = 60)	26.45 ± 6.05	35.13 ± 2.27	25.75 ± 3.58

## Data Availability

The data used to support the findings of this study are available from the corresponding author upon request.

## References

[1] Gariepy A., Lundsberg L. S., Vilardo N., Stanwood N., Yonkers K., Schwarz E. B. (2017). Pregnancy context and women’s health-related quality of life. *Contraception*.

[2] Wilkerson R. G., Ogunbodede A. C. (2019). Hypertensive disorders of pregnancy. *Emergency Medicine Clinics of North America*.

The article "Evaluation of Cardiac Function of Pregnant Women with High Blood Pressure during Gestation Period and Coupling of Hearts with Peripheral Vessels by Ultrasonic Cardiogram under Artificial Intelligence Algorithm" was retracted in 2023. Reasons: signs of a paper mill; compromised peer review; unreliable results or conclusions.

[3] Donoho D. L. (2006). Compressed sensing. *IEEE Transactions on Information Theory*.

[4] Hauspurg A., Countouris M. E., Catov J. M. (2019). Hypertensive disorders of pregnancy and future maternal health: how can the evidence guide postpartum management?. *Current Hypertension Reports*.

[5] Ankumah N. E., Sibai B. M. (2017). Chronic hypertension in pregnancy: diagnosis, management, and outcomes. *Clinical Obstetrics and Gynecology*.

[6] Liu F. M., Zhao M., Wang M., Yang H. L., Li L. (2016). Effect of regular oral intake of aspirin during pregnancy on pregnancy outcome of high-risk pregnancy-induced hypertension syndrome patients. *European Review for Medical and Pharmacological Sciences*.

[7] Silversides C. K., Grewal J., Mason J. (2018). Pregnancy outcomes in women with heart disease: the CARPREG II study. *Journal of the American College of Cardiology*.

[8] Moors S., Staaks K. J., Westerhuis M. E. (2020). Heart rate variability in hypertensive pregnancy disorders: a systematic review. *Pregnancy Hypertens*.

[9] Easter S. R., Rouse C. E., Duarte V. (2020). Planned vaginal delivery and cardiovascular morbidity in pregnant women with heart disease. *American Journal of Obstetrics and Gynecology*.

[10] Mehta L. S., Warnes C. A., Bradley E. (2020). Cardiovascular considerations in caring for pregnant patients: a scientific statement from the American Heart Association. *Circulation*.

[11] Hansen P. R., Isaksen J. L., Jemec G. B., Ellervik C., Kanters J. K. (2018). Ankle-brachial index in psoriasis: a population-based study. *International Journal of Dermatology*.

[12] Lv Z., Chen D., Lou R., Wang Q. (2021). Intelligent edge computing based on machine learning for smart city. *Future Generation Computer Systems*.

[13] Hu M., Zhong Y., Xie S., Lv H., Lv Z. (2021). Fuzzy system based medical image processing for brain disease prediction. *Frontiers in Neuroscience*.

[14] Gojnic M., Pervulov M., Petkovic S. (2004). Early diagnosis of trophoblast produced capillary hypertension (pregnancy-induced hypertension). *Clinical and Experimental Obstetrics & Gynecology*.

[15] Magee L. A., von Dadelszen P. (2018). State-of-the-art diagnosis and treatment of hypertension in pregnancy. *Mayo Clinic Proceedings*.

[16] Saba L., Jamthikar A., Gupta D. (2019). Global perspective on carotid intima-media thickness and plaque: should the current measurement guidelines be revisited?. *International Angiology*.

[17] Nemeth Z., Hildebrandt E., Ryan M. J., Granger J. P., Drummond H. A. (2020). Pressure-induced constriction of the middle cerebral artery is abolished in TrpC6 knockout mice. *American Journal of Physiology-Heart and Circulatory Physiology*.

The article "Evaluation of Cardiac Function of Pregnant Women with High Blood Pressure during Gestation Period and Coupling of Hearts with Peripheral Vessels by Ultrasonic Cardiogram under Artificial Intelligence Algorithm" was retracted in 2023. Reasons: signs of a paper mill; compromised peer review; unreliable results or conclusions.

[18] Hametner B., Wassertheurer S., Mayer C. C., Danninger K., Binder R. K., Weber T. (2021). Aortic pulse wave velocity predicts cardiovascular events and mortality in patients undergoing coronary angiography. *Hypertension*.

[19] Mueller N., Streis J., Müller S. (2020). Pulse wave analysis and pulse wave velocity for fistula assessment. *Kidney & Blood Pressure Research*.

[20] Ma Y., Choi J., Hourlier-Fargette A. (2018). Relation between blood pressure and pulse wave velocity for human arteries. *Proceedings of the National Academy of Sciences*.

[21] Cianci R., Gigante A., Gasperini M. L., Barbano B., Galea N., Rosato E. (2020). Late gadolinium enhancement in cardiac magnetic resonance imaging is associated with high renal resistive index in patients with systemic sclerosis. *Kidney & Blood Pressure Research*.

[22] for the Preterm SAMBA study group, Mayrink J., Souza R. T. (2019). Mean arterial blood pressure: potential predictive tool for preeclampsia in a cohort of healthy nulliparous pregnant women. *BMC Pregnancy Childbirth*.

[23] Potkonjak A. M., Sabolović Rudman S., Nikolac Gabaj N. (2020). Urinary troponin concentration as a marker of cardiac damage in pregnancies complicated with preeclampsia. *Medical Hypotheses*.

[24] Pisani I., Tiralongo G. M., Lo Presti D. (2017). Correlation between maternal body composition and haemodynamic changes in pregnancy: different profiles for different hypertensive disorders. *Pregnancy Hypertension*.

[25] Giorgione V., O'Driscoll J., Coutinho C. M. (2021). Peripartum echocardiographic changes in women with hypertensive disorders of pregnancy. *Ultrasound in Obstetrics & Gynecology*.

[26] Botta L., Merati R., Vignati G. (2016). Mitral valve endocarditis due toAbiotrophia defectivain a 14th week pregnant woman. *Interactive Cardiovascular and Thoracic Surgery*.

